The article "Online Automatic Diagnosis System of Cardiac Arrhythmias Based on MIT-BIH ECG Database" was retracted in 2023. Reasons: signs of a paper mill; suspected computer-generated content; unreliable results or conclusions; concerns about the data.

# Online Automatic Diagnosis System of Cardiac Arrhythmias Based on MIT-BIH ECG Database

**DOI:** 10.1155/2021/1819112

**Published:** 2021-12-16

**Authors:** Wei Yan, Zhen Zhang

**Affiliations:** Department of Cardiovascular Medicine, Affiliated Hospital of Youjiang Medical College for Nationalities, Guangxi, Baise, China

## Abstract

Arrhythmias are a relatively common type of cardiovascular disease. Most cardiovascular diseases are often accompanied by arrhythmias. In clinical practice, an electrocardiogram (ECG) can be used as a primary diagnostic tool for cardiac activity and is commonly used to detect arrhythmias. Based on the hidden and sudden nature of the MIT-BIH ECG database signal and the small-signal amplitude, this paper constructs a hybrid model for the temporal correlation characteristics of the MIT-BIH ECG database data, to learn the deep-seated essential features of the target data, combine the characteristics of the information processing mechanism of the arrhythmia online automatic diagnosis system, and automatically extract the spatial features and temporal characteristics of the diagnostic data. First, a combination of median filter and bandstop filter is used to preprocess the data in the ECG database with individual differences in ECG waveforms, and there are problems of feature inaccuracy and useful feature omission which cannot effectively extract the features implied behind the massive ECG signals. Its diagnostic algorithm integrates feature extraction and classification into one, which avoids some bias in the feature extraction process and provides a new idea for the automatic diagnosis of cardiovascular diseases. To address the problem of feature importance variability in the temporal data of the MIT-BIH ECG database, a hybrid model is constructed by introducing algorithms in deep neural networks, which can enhance its diagnostic efficiency.

## 1. Introduction

Cardiac diseases are the deadliest chronic diseases and are characterized by high morbidity, disability, and mortality. Nowadays, the prevalence and mortality of cardiovascular diseases are still on the rise worldwide [1]. Electrocardiogram (ECG) is the main diagnostic tool for CVD in clinical practice and is commonly used to detect cardiac arrhythmias. Arrhythmias are a common and complex cardiovascular disease that usually precedes the onset of arrhythmias. Early detection allows for appropriate intervention and thus can reduce unnecessary disability and death in the early stages of cardiovascular disease. ECG signals are insidious and abrupt, making it difficult to provide a comprehensive and accurate picture of a patient's cardiac status. Holter generates a large amount of ECG data, but the current manual ECG signal analysis is limited in real-time and accuracy [2]. Currently, physicians mainly use post hoc analysis to determine whether a patient is ill and the possible type of disease through waveform analysis, which is time-consuming, inefficient, and not highly reliable due to factors such as physician expertise and experience level. Physicians are unable to complete real-time online analysis of large-scale ECG data. Computer-aided analysis based on ECG can effectively improve medical diagnosis efficiency and shorten diagnosis time and has reliable clinical application value. The basis of automatic analysis technology of ECG data is to effectively extract features and then use a priori knowledge or machine learning methods to classify and diagnose. A priori knowledge comes from doctors' clinical experience, and ECG algorithms have limitations in P wave and T-wave recognition and cannot analyze their bands as a complete wave group [3]. Traditional automatic analysis methods of machine learning often use shallow neural networks to classify and identify ECG data waveform features, which can automatically adjust parameters and cover multiple features, with limited nonlinear fitting and approximation capabilities in the face of complex classified ECG data. In the context of big data-driven training, the recognition efficiency of shallow neural network classifiers is not high for big data training; in addition, the nonlinear fitting ability and accuracy are limited. Deep learning fuses feature extraction and classification, which is beneficial to improve recognition rates. However, deep neural networks deepen the difficulty of training optimization as the number of layers deepens, and the models lack strong interpretability. Under the condition of massive ECG data, traditional feature extraction cannot effectively extract the deep essential features of the target data, and how to automatically analyze and explore the potential value becomes an important opportunity and challenge in the field of ECG. Aiming at remote ECG monitoring, the core key issues in waveform features that distinguish it from the traditional ones are addressed by designing and implementing a remote ECG monitoring system. Conducting research on data-driven and deep learning-based intelligent classification and identification of cardiac arrhythmias and proposing convenient and feasible methods for self-diagnosis of cardiovascular diseases are of great practical significance for economic and social development and people's health [4].

The article "Online Automatic Diagnosis System of Cardiac Arrhythmias Based on MIT-BIH ECG Database" was retracted in 2023. Reasons: signs of a paper mill; suspected computer-generated content; unreliable results or conclusions; concerns about the data.

ECG diagnosis is currently done mainly by manual analysis, but in today's world where cardiovascular diseases are generally high, an extremely large amount of ECG data is generated every day and every hour, and the types of heartbeats are very diverse, so manual management and analysis of ECG on a beat-by-beat basis is a task that is difficult to accomplish effectively. Especially in a clinical monitoring or wearable health monitoring environment, real-time diagnosis is even more of an unachievable task for healthcare staff due to the lack of expert resources for ECG diagnosis and high labor intensity. In addition, the suddenness and infrequency of the appearance of some abnormal heartbeats make it difficult for cardiologists to capture some important changes in an emergency condition promptly, which will directly threaten the life safety of patients. How to automatically and timely identify abnormal heartbeats from a large amount of ECG data and improve the accuracy and timeliness of ECG diagnosis is an important and necessary task. ECG automatic diagnosis technology can reduce the labor intensity of ECG specialists, eliminate misdiagnosis and misdiagnosis caused by subjective factors of medical personnel, and thus improve monitoring and diagnosis. The ECG automatic diagnosis system can be embedded into wearable devices (bracelets, medical vests, etc.) to provide long-term real-time monitoring of cardiac conditions, enhance prevention and thus timely detect heartbeat abnormalities, buy valuable time for further treatment of patients, provide favorable conditions, reduce medical costs, and ease the burden on patients, thus increasing the cure rate of cardiovascular diseases. Therefore, the research of ECG automatic diagnosis technology has an important role in promoting the progress of medicine and is of great significance in solving the current problems in ECG diagnosis.

## 2. Related Work

Automatic diagnosis of ECG is one of the hot spots in the field of ECG research, especially in the field of real-time diagnosis of ECG signals [5]. The variability of heartbeat waveforms in various heart disease patients and the fact that the recording devices of heartbeat signals are often influenced by the working environment and introduce a large number of different types of noise information make the effective diagnosis of ECG very difficult, and it is still a challenging research problem. Various methods have emerged in the area of heartbeat recognition, which is broadly classified into supervised and unsupervised methods. Supervised recognition methods are recognition algorithms that are constructed based on data with labels. The representative methods are convolutional neural networks [6], radial basis neural networks, least squares support vector machines, and so on. Unsupervised recognition methods refer to recognition algorithms constructed based on data with labels, and representative methods are self-coding neural networks [7], K-means clustering algorithms, and so on. Among them, the literature uses a convolutional neural network model to identify the heartbeat of a specific patient for the specificity between different patients. The method takes into account the blind spots in the diagnosis of new patients and provides a new idea for the automatic diagnosis of ECG. After this feature learning phase [8], the algorithm adds a softmax classification layer on top of the generated hidden representation layer to generate a deep neural network (DNN). The DNN model is then used to identify the heartbeat. This method can reduce the expert interaction to some extent. A deep learning-based method for single-lead ECG signal classification was proposed by literature. The method is an application of finite Boltzmann machine (RBM) and deep confidence network (DBN) for ECG classification after detection of ventricular and supraventricular heartbeats in single-lead ECG. The algorithm is validated using the MIT-BIH ECG database at a low sampling rate of 114 HZ. The RBM and DBN are selected with appropriate parameters, and higher performance can be obtained for heartbeat recognition, and it achieves better recognition results at a lower sampling rate compared to conventional methods [9].

The article "Online Automatic Diagnosis System of Cardiac Arrhythmias Based on MIT-BIH ECG Database" was retracted in 2023. Reasons: signs of a paper mill; suspected computer-generated content; unreliable results or conclusions; concerns about the data.

The literature uses a five-level discrete wavelet transform to decompose the signal into six subband signals with different frequency distributions. Three RR interval correlation features were added to construct a feature vector of 30 features, and finally [10] the features were fed into a feedforward backpropagation neural network to achieve the classification of seven signals. Transformation extracted wavelet coefficients of ECG signals as the first features and optimized the wavelet extracted features using a combination of principal component analysis and independent component analysis and then fused intervals as the final features. Finally, the classification of six classes of ECG signals was achieved in the classifier and achieved 96.31% accuracy [11]. The literature uses geometric positions on the phase curve to extract ECG signal features from the detected R-peaks. Finally, the extracted features were fed into a support vector machine and K-neighborhood to achieve normal and abnormal signal classification [12]. The literature used the first-order derivative of Gaussian function as wavelet basis function and ECG feature extraction by examining the position of the modal maximal pair in the corresponding level of wavelet transform as a range for searching R-wave vertices in QRS waves, thus achieving 93% accuracy of abnormal heart rate in MIT-BIH database. The literature et al. used discrete wavelet transform combined with three-dimensionality reduction methods, principal component analysis, linear discriminant analysis, and ICA [13] and sent the reduced features to SVM, neural network, and probabilistic neural network classifier to achieve the automatic classification of a total of five ECG signals, namely, nonheterodyne beats, supraventricular heterodyne beats, ventricular heterodyne beats, fused heartbeats, and paced heartbeats. The contribution uses Harr wavelet transform to extract features from ECG signals. Feedforward neural network was used for preprocessing and classification of ECG signals. Classification of left bundle branch block, right bundle branch block, premature ventricular beats, premature atrial beats, premature lymph node beats, and normal beats was implemented in the MIT-BIH database [14].

The article "Online Automatic Diagnosis System of Cardiac Arrhythmias Based on MIT-BIH ECG Database" was retracted in 2023. Reasons: signs of a paper mill; suspected computer-generated content; unreliable results or conclusions; concerns about the data.

## 3. MIT-BIH Cardiac Database for Online Automatic Diagnosis of Cardiac Arrhythmias

### 3.1. MIT-BIH ECG Database

The ECG signal is an electrical signal generated by the movement of the heart measured from the surface of the human body by an instrument. In the process of obtaining the ECG signal, there are inevitably many interfering factors, such as the instrument and the environment. These interferences will alter the true ECG signal. These interferences will alter the real human ECG signal, which is the basis for doctors to diagnose heart diseases, and any interference will cause misdiagnosis [15], thus causing irreparable harm to the patient. For the researcher, the noise generated by the interference will affect the results of the study. The MIT-BIH ECG data collected under different devices and different environmental conditions can interfere with the real signal to different degrees due to various interference factors, and we call the data in the MIT-BIH database heterogeneous data. To reduce or even avoid the harm caused by noise, the main work in this section is the study of MIT-BIH ECG databases, by perfecting the preprocessing methods so that MIT-BIH data can be cross-used [16], each MIT-BIH ECG database has its characteristics, such as the number of leads, storage format, and sampling frequency, but the common purpose is to conduct research or perform disease diagnosis. The principle of the formula lies in

(1) $$\begin{array}{c} A=\sum_{i=1}^{n}X_{i}Y_{i}+\sum_{i=1}^{n}X_{i}Y_{i}. \end{array}$$

Formula (1) plays an important role in the construction of the database in the article. It can ensure the normal operation of the database and ensure that there is enough storage space. This is its role and can help the normal operation of the entire system. Currently, there are many ECG databases, but there is no single standard, and researchers can only analyze one ECG database for their research and cannot use others, which is a great waste of resources. For research analysis in cardiac diseases, adequate data is an important guarantee for the sustainability of the research. In addition to the number of leads and storage formats, the different sampling frequencies and signal quality of the MIT-BIH ECG databases are also obstacles to cross-use between the MIT-BIH ECG databases. The concept of big data is now known and valued by more and more researchers, entrepreneurs, companies, etc., and can be used to fully exploit the correlations and useful information in huge data sets using advanced algorithms, which can then be applied in practice to bring greater value to people, with data algorithms as

(2) $$\begin{array}{c} T=\frac{\Delta y}{\Delta x}.\frac{\delta y}{\delta x}.\frac{\partial^{2}\Omega }{\partial u\;\partial v}. \end{array}$$

The function of formula (2) has a connecting effect on the paper. For the structure of the paper, formula (1) can be further described, or a series of introductions can be made to the following content to optimize the structure of this chapter. It is also true for ECG database, data is money, how to make full use of the existing database, how to remove the barriers between MIT-BIH ECG databases and facilitate the cross-use between MIT-BIH databases, these studies are very valuable. The ECG database is the first database for the Chinese population, containing 11 major categories of ECG abnormalities and 100+ categories of subdivided ECG symptoms, with data types including conventional ECG, single-lead, 3-5-lead, and 12-lead ECG. In the form of data presentation, each ECG data contains data source, recording time, length, ECG plot, analysis of various indexes, and expert labeling. At the same time, each ECG data records patient age, gender, disease information, and so on. The database covers a wider range of ECG abnormality types and richer data types, which can provide shared services and technical support for related institutions and significantly reduce the R&D cost. The traditional encoder is shown in Figure 1.

The article "Online Automatic Diagnosis System of Cardiac Arrhythmias Based on MIT-BIH ECG Database" was retracted in 2023. Reasons: signs of a paper mill; suspected computer-generated content; unreliable results or conclusions; concerns about the data.

To verify the effectiveness of the above combination of denoising methods on heterogeneous data, preprocessing was performed, followed by a detailed similarity comparison. PTB is a German diagnostic ECG database. PTB is a German diagnostic ECG database containing 549 records from 290 individuals with 15 lead signal records per individual in the conventional 12 leads (i, ii, iii v1, v2, v3, v4, v5, and v6) and 3 Frank leads (vx, vy, and vz) with a sampling frequency of 1000 Hz, containing a wide range of disease samples and healthy comparison samples; VGHTC is an ECG database from Taichung Veterans General Hospital, containing tens of thousands of cases, each with a conventional 12-lead ECG signal with a sampling frequency of MIT-BIH being a self-collected ECG database containing 30 individual samples with a two-lead approach and a sampling frequency of 250 Hz, and due to the limitations, the samples in this database are all healthy samples. Since the samples in each heterogeneous ECG database have different types of diseases but all contain healthy samples, the healthy samples from the three databases were chosen for this experiment to ensure the consistency of the experimental data [17]. Left bundle branch conduction block, also known as left bundle branch block, results from delayed conduction of electrical excitation in the left bundle branch of the heart or interrupted; the excitation can only be transmitted from the right to the left ventricle of the heart, resulting in some delay in the excitation of the left ventricle. Right bundle branch conduction block is caused by a block in the right bundle branch of the heart, which in turn causes electrical excitation to fail via the pathway into the right ventricle and must be signaled by signals from the left ventricle [18]. However, the electrical signals from the left ventricle must pass through myocardial afferents, and this pathway is transmitted more slowly than the original Hitchcock–Purkinje fiber pathway, so on the ECG, the patient will have a wider complex wave. Also, because the left ventricle depolarizes faster than the right ventricles and therefore in the wave will produce a condition where the heart axis is offset, atrial preterm contraction is also known as atrial premature beat. It is a single or paired ectopic atrial excitation that originates anywhere in the atria other than the sinus node. In the presence of atrial premature beats, the P wave is distinctly different from the normal sinus P wave, and the time frame of the P-R interval is generally outside the normal range. Ventricular contractions, or premature ventricular contractions, are a premature excitation of the ventricles due to various causes. The arrhythmia can occur in patients of any age with cardiovascular disease and the general population. In the ECG signal, abnormally wide wave clusters are observable, and there is an inversion of the T-wave following the QRS wave cluster. Pacemaker rhythm is the rhythm produced by controlling the heartbeat with external electrical stimulation when sinus bradycardia, sinus arrest, and simultaneous block of the right and left bundle branches of the AV node result in severe ventricular rate slowing that is unable to maintain the body's physiological needs. Due to different clinical needs, the pacemaker program control mode is set differently, and the human autonomic rhythm often coordinates with the pacing rhythm to control the heartbeat, making the pacing ECG variable and a difficult clinical diagnosis. The types of pacing are divided into atrial pacing, ventricular pacing, three-chamber pacing, and four-chamber pacing, depending on the location. In most cases, arrhythmias are unconditioned, and they occasionally occur in normal individuals. However, frequent arrhythmias are usually caused by cardiovascular disease, and therefore the diagnosis of arrhythmias is important for the prevention of cardiovascular disease.

The article "Online Automatic Diagnosis System of Cardiac Arrhythmias Based on MIT-BIH ECG Database" was retracted in 2023. Reasons: signs of a paper mill; suspected computer-generated content; unreliable results or conclusions; concerns about the data.

### 3.2. MIT-BIH Arrhythmia Online Automatic Diagnosis System

The MIT-BIH Arrhythmia Database is MIT's international standard-based, expertly diagnosed, and annotated ECG database, and the standard ECG database is widely recognized and used in academia. The database in this paper is an important source of data for the research work on automatic arrhythmia diagnosis algorithm. The MIT-BIH arrhythmia database has more than a dozen types of arrhythmias, totaling more than 100,000 heartbeats, excluding most of the normal beats, among which are atrial premature beats, ventricular premature beats, bundle branch block, atrial fibrillation, and many other types of abnormal heartbeats. The database provides a uniform naming of the various arrhythmias. For ease of annotation, each beat is marked with a special symbol. Arrhythmias are abnormalities in the frequency, rhythm, origin, conduction velocity, and sequence of excitation of the electrical impulses of the heart, with the direct consequence of sudden cardiac death and heart failure [19]. It is estimated that there are hundreds of millions of cardiovascular patients worldwide, of whom 26.8% suffer from arrhythmias, and the prevalence and mortality rates are still on the rise. Currently, various imaging techniques, electrocardiograms, and electrocardiogram imaging are available for the diagnosis of arrhythmias, and treatments include antiarrhythmic drugs, artificial pacemakers, heart transplants, cardiac stents, heart bypasses, radiofrequency ablation, and so on. Although advanced treatment techniques and drugs have reduced the death rate of arrhythmias, some treatment modalities (such as antiarrhythmic drugs and radiofrequency ablation) have not only failed to cure arrhythmias but also become the key factors leading to arrhythmias, making the death rate of arrhythmias remain high. Despite the rapid development of modern medical technology, the incidence of arrhythmias remains high. Taking atrial fibrillation as an example, ECG is still the core method of arrhythmia diagnosis. Traditional arrhythmia diagnosis relies on ambulatory electrocardiography (Holter) to provide 24 h ECG monitoring. Patients carry continuous ECG information with them. The need for patients to carry instruments, leads, and spacers with them to use the Holter is extremely uncomfortable and disruptive, and the subsequent data processing is cumbersome, limiting its use on a large scale, while short-duration 12-lead ECGs often lead to missed arrhythmias. ECG signals are low-frequency and weak electrical signals collected from the human body surface by ECG monitoring equipment through multiple electrodes. The amplitude of ECG signals is usually in the millivolt range, which is very low, and the signal frequency is usually in the range of 0.05–100 Hz, which is in the low-frequency band. Moreover, the ECG signal may fluctuate due to the difference between the human body and monitoring equipment. Due to the weak characteristics and instability of ECG signals, ECG signals are extremely vulnerable to the influence of external noise. As can be seen from the noise sources, ECG interference is mainly divided into three main categories: one is the industrial frequency interference brought by the circuit equipment; the second is the electromyographic interference brought by the human skin and muscles at the electrode acquisition position; the third is the baseline drift caused by the human body movement or electrode movement and other large changes in position. Industrial frequency interference is the signal acquisition process. The interference signal is generated by the influence of the circuit system. Currently, the domestic frequency of industrial frequency interference is 50 Hz. Industrial frequency interference is the most common and unavoidable interference in the ECG signal, and the maximum amplitude of interference can reach about 50% of the normal ECG signal amplitude. Because the frequency of the IDF interference does not change much, it is usually evident in the ECG. Baseline drift occurs when the ECG signal fluctuates up and down frequently, resulting in a baseline that cannot be maintained at the same level. The main cause of baseline drift is movement during signal acquisition, including the movement of the body and movement of the equipment. Baseline drift is extremely common in 24-hour ECGs. Baseline drift can severely affect the amplitude of the ECG signal, making it impossible to calculate the exact amplitude of individual waveforms from a baseline position, which in turn can affect the diagnosis of disease.  Figure 2 shows the neural network structure.

The article "Online Automatic Diagnosis System of Cardiac Arrhythmias Based on MIT-BIH ECG Database" was retracted in 2023. Reasons: signs of a paper mill; suspected computer-generated content; unreliable results or conclusions; concerns about the data.

Wavelet transform (WT) is a mathematical transformation method proposed and popularized at the end of the last century. Wavelet transform can maximize the local characteristics of the signal through mathematical transformation and realize time-frequency localization analysis. The mathematical transform is used to decompose the signal data on multiple scales, to process the high and low frequencies of the signal separately [20], to satisfy the adaptive analysis of various frequencies, and then to realize the local analysis of any part of the signal, which overcomes the difficult problem of Fourier transform in signal processing. Wavelets are obtained from fundamental wavelets by mathematical transformation “stretching translation”. The fundamental wavelet is a function with fast decay properties, and this function needs to mathematically satisfy the requirement of zero integration:

(3) $$\begin{array}{c} M=\sum_{i=1}^{n}X_{i}Y_{i}+\frac{1}{n}\left(\frac{x-\mu }{\sigma }\right). \end{array}$$

Wavelet transform has the following good properties: (1) low entropy: due to the sparse nature of the WT coefficient distribution, the entropy of the signal after processing becomes very low; (2) multiresolution characteristics: wavelet transform can be a multiscale transform for processing local details, which can well retain the nonsmooth characteristics of the signal; (3) decorrelation: after the ECG signal is transformed by wavelet, the noise signal in it tends to be whitened, so it is easier to distinguish the two, making the wavelet; (4) flexibility of base selection: due to the diversity of wavelet basis functions, the wavelet transform method is more flexible in processing different signal data, so more suitable wavelet basis functions can be selected to improve the signal processing effect.

After wavelet decomposition of the ECG signal acquired by the device, the key features of the human ECG signal tend to be distributed and are on wavelet coefficients of high amplitude, while wavelet coefficients of smaller amplitude mostly contain various useless noises, while wavelet decomposition can also be corrected for the baseline drift of the signal. This topic is addressed by setting the signal with the original. Strongly correlated adaptive thresholds are used to zero out wavelet coefficients that are smaller than the threshold so that the ECG signal is the purpose of denoising. The main process is divided into three steps as shown in Figure 3.

Scale wavelet decomposition is as follows. Select a wavelet and determine the level of decomposition, and then carry out the decomposition calculation. Wavelet threshold processing is as follows. According to the signal-to-noise ratio of the original signal and the decomposed high-frequency coefficients, calculate the threshold value associated with it, screen the noise information by the threshold value, and then carry out quantization processing. Wavelet coefficient reconstruction is as follows. The decomposed wavelet coefficients are retransformed to a one-dimensional wavelet reconstruction. In the whole process, the selection of wavelet basis, the determination of decomposition scale, and the setting of threshold are the key to the wavelet denoising process, which will directly affect the effectiveness of the signal after reconstruction. In signal processing, usually, these three key parameters do not have a fixed selection method. For different signals, the best experimental parameters need to be selected and experimented with according to the characteristics of the signal, the characteristics of the noise, and the actual needs. The improved wavelet filtering process is shown in Figure 4.

The article "Online Automatic Diagnosis System of Cardiac Arrhythmias Based on MIT-BIH ECG Database" was retracted in 2023. Reasons: signs of a paper mill; suspected computer-generated content; unreliable results or conclusions; concerns about the data.

## 4. Experimental Results and Analysis

### 4.1. Experimental Results

The features extracted from the heartbeat waveform are mainly time-domain features and voltage amplitude features, and obtaining the main features has an important connection with the number of convolutional kernels. To investigate the effect of the number of convolutional kernels on the accuracy of the test set in the CNN model, this paper keeps the learning rate and training times constant and adjusts the number of convolutional kernels to observe the change in the accuracy of the test set with the number of network layers as 2. During the experiment, it is found that the time spent on training samples is positively related to the number of convolutional kernels. By comparison, it can be found that the number of convolutional kernels is more realistic when the number of convolutional kernels is 5. After the training is completed, the test set heartbeat data is used for testing, and the results obtained from the experiments are compared with the heart expert labeling results to construct a 1D CNN structure validation for heartbeats, which can obtain higher results for classifier performance evaluation metrics. To reflect the obvious advantage of 1D CNN network structure in the classification effect, a comparison test with the classical classifier SVM is performed. The coefficients of the wavelet transform are used as features of the classifier SVM, and its comparative efficiency graph is shown in Figure 5.

In this chapter, the ECG signal in the first channel of 119.dat in MIT-BIH data is selected to verify the filtering algorithm by extending the intercepted signal and adding a constant value to each sampling point in the signal, so that the S-T segment and P-T segment of the signal coincide with the baseline of the zero potential point, and, finally, the ECG signal will be considered pure without baseline drift interference, that is, signal S, where the horizontal coordinate is the number of sampling points, and the vertical coordinate is the voltage value/mV. The baseline drift noise is selected as the signal BW within the second channel of the baseline drift noise bw.dat in MIT-BIH, as shown in Figure 6, which is a plot of the number of experiments and the recognition rate.

The article "Online Automatic Diagnosis System of Cardiac Arrhythmias Based on MIT-BIH ECG Database" was retracted in 2023. Reasons: signs of a paper mill; suspected computer-generated content; unreliable results or conclusions; concerns about the data.

To select a more effective feature extraction method, three feature extraction methods, wavelet feature extraction, improved RBP algorithm, and waveform features described earlier are applied to practical classification, and the classification results are compared in this paper. For the improved RBP features, 36 sets of experiments are conducted based on the parameters m-bit and interval, and the highest recognition rate is taken here. The average recognition rates achieved by the improved wavelet features and the improved RBP algorithm on the proposed multiorder classification algorithm are 78.8% and 64.5%, respectively. The efficiency of the three approaches is compared as shown in Figure 7.

However, often the recognition of one of the classes of heartbeats is not very good, resulting in being poor overall. Of course, there are also good classification results, like MSE, NSE + MSE, MSE + RMSE, and NSE + MSE + RMSE. These feature sets have good classification results. It is observed that the MSE feature set is included in the above feature set, which indicates that the MSE feature set is more effective in classifying the heartbeats of this database. The last row of the table lists the multiorder classification recognition rate of this paper, and by comparison, it is found that although not every heartbeat has a higher recognition rate, the average recognition rate is higher than the other schemes, and it has a better recognition effect for every class of heartbeats as shown in Figure 8. Its representation shows the graph of its efficiency.

## 5. Conclusion

Cardiovascular diseases seriously damage the physical and mental health of the population and have a great impact on people's normal life. Therefore, it is important to prevent the occurrence of cardiovascular diseases in advance in daily life and to perform ECG examinations regularly. At the present stage, the diagnostic method of ECG still relies on the professional physician to implement the diagnosis using the observation method and this transmission. The conventional method consumes a lot of human and material resources and also greatly wastes the precious treatment time of doctors and patients, because it is particularly important to design an automated arrhythmia detection algorithm. Currently, some cardiac monitoring devices propose provided basic arrhythmia methods, but due to the different devices from different manufacturers and the poor immunity of some devices to interference, The diagnostic accuracy of arrhythmias is limited and there is no uniform algorithm that can identify all device signals. In recent years, as deep learning models have made good progress in various fields, they have been used to deal with some prediction and subclass of problems when obtaining high accuracy, as this paper combines deep learning methods and proposes a deep learning method based on degrees of learning in the diagnosis of arrhythmias.

The article "Online Automatic Diagnosis System of Cardiac Arrhythmias Based on MIT-BIH ECG Database" was retracted in 2023. Reasons: signs of a paper mill; suspected computer-generated content; unreliable results or conclusions; concerns about the data.

The main data source for this research work is the MIT-BIH arrhythmia database. The MIT-BIH arrhythmia database is also one of the authoritative databases recognized by the current academic community. This database uses a standard data storage format, and all data have been labeled by professional physicians, which is a reliable data source for model training. Soft thresholding filtering method is based on wavelet decomposition. Wavelet decomposition can transform the signal through time frequency, which can eliminate both high-frequency noise and baseline drift in the ECG signal. With the adaptive soft thresholding method, the eliminated noise can be fine-tuned according to the signal-to-noise ratio of the signal to prevent the normal waveform from being affected.

## Figures and Tables

**Figure 1:** Conventional self-encoder structure.

**Figure 2:** Algorithm model framework diagram.

**Figure 3:** Wavelet filtering flow.

**Figure 4:** Improved wavelet filtering process.

**Figure 5:** Efficiency comparison chart.

**Figure 6:** Number of experiments versus efficiency experimental analysis.

**Figure 7:** Comparison of the efficiency of the three approaches.

**Figure 8:** Electrocardiographic efficiency plot for the MIT-BIH approach.

## Data Availability

The data used to support the findings of this study are available from the corresponding author upon request.

## References

[1] Trayanova N. A., Popescu D. M., Shade J. K. (2021). Machine learning in arrhythmia and electrophysiology. *Circulation Research*.

[2] Herrmann J. (2020). Adverse cardiac effects of cancer therapies: cardiotoxicity and arrhythmia. *Nature Reviews Cardiology*.

[3] Mattioli A. V., Ballerini Puviani M., Malagoli A. (2020). Quarantine and Isolation during COVID‐19 outbreak: a case of online diagnosis of supraventricular arrhythmia through telemedicine. *Journal of Arrhythmia*.

The article "Online Automatic Diagnosis System of Cardiac Arrhythmias Based on MIT-BIH ECG Database" was retracted in 2023. Reasons: signs of a paper mill; suspected computer-generated content; unreliable results or conclusions; concerns about the data.

[4] Singh M., Rao R., Gupta S. (2020). Kardia mobile for ECG monitoring and arrhythmia diagnosis. *American Family Physician*.

[5] Gupta A., Lokhandwala Y., Rai N., Malviya A. (2021). Adenosine-A drug with myriad utility in the diagnosis and treatment of arrhythmias. *Journal of Arrhythmia*.

[6] Pranata R., Chintya V., Raharjo S. B., Yamin M., Yuniadi Y. (2020). Longer diagnosis‐to‐ablation time is associated with recurrence of atrial fibrillation after catheter ablation-Systematic review and meta‐analysis. *Journal of arrhythmia*.

[7] Dewi I. P., Dharmadjati B. B. (2020). Short QT syndrome: the current evidences of diagnosis and management. *Journal of Arrhythmia*.

[8] Claus I., Adriaenssens B., Van Beeumen K., Timmers L., Bové T. (2020). Congenital left ventricular diverticulum: a rare cause of cardiac arrhythmia. *Journal of Cardiac Surgery*.

[9] Islam M. S., Alajlan N. (2018). Model-based alignment of heartbeat morphology for enhancing human recognition capability. *Computer Journal*.

[10] Nair M., Bhagirath P., Gothi R. (2020). Life‐threatening ventricular arrhythmia as first presentation of tuberculosis-early diagnosis and successful treatment: a case series. *Pacing and Clinical Electrophysiology*.

[11] Gupta V., Mittal M. (2020). A novel method of cardiac arrhythmia detection in electrocardiogram signal. *International Journal of Medical Engineering and Informatics*.

[12] Liu Y., Wu W. (2020). Cardiovascular immune‐related adverse events: evaluation, diagnosis and management. *Asia-Pacific Journal of Clinical Oncology*.

[13] Sulaiman S., Yousef N., Benjamin M. M. (2020). Burden of arrhythmia and electrophysiologic procedures in alcoholic cardiomyopathy hospitalizations. *International Journal of Cardiology*.

[14] Karboub K., Tabaa M., Monteiro F., Dellagi S., Moutaouakkil F., Dandache A. (2020). Automated diagnosis system for outpatients and inpatients with cardiovascular diseases. *IEEE Sensors Journal*.

[15] Huang Y., Liu H., Wu C. (2021). Ventricular arrhythmia predicts poor outcome in polymyositis/dermatomyositis with myocardial involvement. *Rheumatology*.

[16] Cheikhrouhou O., Mahmud R., Zouari R., Ibrahim M., Zaguia A., Gia T. N. (2021). One-dimensional CNN approach for ECG arrhythmia analysis in fog-cloud environments. *IEEE Access*.

[17] Rashed-Al-Mahfuz M., Moni M. A., Lio’ P. (2021). Deep convolutional neural networks based ECG beats classification to diagnose cardiovascular conditions. *Biomedical engineering letters*.

[18] Costa R., Winkert T., Manhães A., Teixeira J. P. (2021). QRS peaks, P and T waves identification in ECG. *Procedia Computer Science*.

The article "Online Automatic Diagnosis System of Cardiac Arrhythmias Based on MIT-BIH ECG Database" was retracted in 2023. Reasons: signs of a paper mill; suspected computer-generated content; unreliable results or conclusions; concerns about the data.

[19] Ahmad Z., Tabassum A., Guan L., Khan N. M. (2021). ECG heartbeat classification using multimodal fusion. *IEEE Access*.

[20] Pandeyz S. K., Janghel R. R., Gupta V. (2021). Cardiac arrhythmia detection and classification from ECG signals using XGBoost classifier. *Machine Learning Algorithms and Applications*.

